# Effect of Comprehensive Nursing on Traumatic Paraplegia Patients by Evaluation of Magnetic Resonance Imaging Features

**DOI:** 10.1155/2022/4712797

**Published:** 2022-08-29

**Authors:** Rui Xiang, Fengqin Xu, Zhaoyang Yin, Lili Ji, Qin Xu

**Affiliations:** ^1^Department of Orthopedics, Lianyungang Clinical College of Nanjing Medical University, The First People's Hospital of Lianyungang, Lianyungang 222061, Jiangsu, China; ^2^Nursing Department, Lianyungang Clinical College of Nanjing Medical University, The First People's Hospital of Lianyungang, Lianyungang 222061, Jiangsu, China; ^3^School of Nursing, Nanjing Medical University, Nanjing 211166, Jiangsu, China

## Abstract

This research aimed to discuss the comprehensive nursing under the Omaha system in the treatment of patients with traumatic paraplegia (TP) and the changes in magnetic resonance imaging (MRI) features of patients. In total, 60 patients with TP were included as the research objects, and they were randomly divided into the experimental group (Omaha system-based comprehensive nursing) and the control group (routine nursing). All the objects underwent parallel MRI multisequence scanning. The scores of the quality of life, role change, mental health, care, oral hygiene, skin, neuromusculoskeletal (NMS) system, defecation function, urination function, contagion/infection, nutrition, healthcare supervision, and rest/sleep pattern in the experimental group were all significantly higher than those in the control group 3 months and 6 months after discharge (*P* < 0.05). The caregiving burden scores in the experimental group 3 months and 6 months after discharge from the hospital were 48.67 ± 6.97 and 43.40 ± 4.97, respectively, statistically lower than those in the control group (52.83 ± 6.37; 50.07 ± 7.14) (*P* < 0.05). On admission, MRI showed that the white lines disappeared from the compression of the dural sac, the spinal cord was compressed, and the intramedullary signal was abnormal. Then, six months after discharge, MRI showed that the compression of the dural sac was relieved, and the double white lines recovered. The apparent diffusion coefficient (ADC) of patients in the experimental group 6 months after discharge (1.063 ± 0.148) was highly lower than that in the control group (1.325 ± 0.245), with a difference of statistical significance (*P* < 0.05). In conclusion, comprehensive nursing under the Omaha system could improve the clinical treatment effect of patients with spinal cord injury (SCI) effectively, reduce the incidence of complications, and improve the quality of life and nursing outcomes of patients.

## 1. Introduction

Traumatic paraplegia (TP) refers to a condition in which the limbs below the position of spinal cord injury (SCI) are paralyzed due to external force on the spine, with perceptual dysfunction and bowel and urine dysfunction [1]. It is mostly caused by direct or indirect violence. The incidence is the highest occurrence in the cervical spine, followed by the thoracic and lumbar segments; the severity of SCI is generally proportional to the magnitude of the violence [2, 3]. TP is one of the most difficult diseases medically today. After the onset, the treatment for SCI by western medicine can only restore the caliber of the spinal canal through surgical decompression so that the patients' life will not be threatened and they will not suffer from permanent paralysis or paraplegia for the damaged spinal cord will not be damaged again [4]. But there is no way to recover the paralyzed nerve after nerve injury, so most patients spend their time in a wheelchair forever. If the ischemic nerve is damaged secondarily due to improper treatment or delayed treatment, the disabled patients will suffer from various comorbidities and will have a very painful life [5–7].

TP has a great impact on patients and their families. How to help patients improve their quality of life and reduce social and family pressure are the focus of current research [8, 9]. Clinical nursing intervention for TP is multifaceted, and comprehensive nursing is very important for patients. Since patients will have anxiety, fear, and pessimism that affect their recovery, it is necessary to encourage patients to build confidence in beating the disease. In terms of nutrition, patients need to be given a high-protein, high-energy, and high-vitamin diet. Patients should be encouraged to breathe deeply, cough, and expectorate sputum to prevent lung infection, etc. For the loss of part of the somatic motor function, muscle atrophy, flexion contracture, foot drop, etc. are prone to occur, and it is necessary to help patients with frequent passive limb training [10]. Generally speaking, most paraplegic patients can achieve the goal of self-care and reintegration into society through medical treatment and functional training. High paraplegic patients cannot stand with crutches due to the affected mobility of all their limbs, so they should be trained to use wheelchairs [11–13]. X-ray is a common method for diagnosing the severity of SCI in patients in recent years. It can display the morphological changes, displacements, and conditions of the spinal canal of the compressed vertebral body, but it still has certain limitations [14]. Magnetic resonance imaging (MRI) distinguishes different tissues, including tumor tissues and normal tissues, according to the signal differences of protons in different compounds. It has been applied in the imaging diagnosis of various systems in the whole body, and it also has a very eye-catching performance in the diagnosis of SCI. MRI has the advantages of no ionizing radiation, multisequence and multidirectional imaging, and high resolution [15].

To sum up, the nursing and treatment of TP still need continuous exploration. Therefore, 60 patients with TP were divided into 30 cases in the experimental group and 30 cases in the control group according to different nursing programs. Comprehensive nursing under the Omaha system was given to the former, while routine nursing was for the latter. All these patients underwent MRI multisequence scanning. By comparing the scores of quality of life, caregiving burden, physiological domain, psychological domain, environmental domain, social health domain, complications, and MRI features of patients before and after the intervention, the application value of the Omaha system-based comprehensive nursing was comprehensively evaluated in the treatment of TP patients.

## 2. Materials and Methods

### 2.1. Research Objects

Sixty patients with TP admitted to the hospital from January to December 2021 were chosen as the research objects, including 38 males and 22 females. Their average age was 35.72 ± 3.14 years old, with an age range of 20–70 years old. They were randomly divided into 30 cases in the experimental group and the other 30 cases in the control group. This research had been approved by the ethics committee of the hospital; the patients and their families were informed about the research and signed the informed consent.

Inclusion criteria included patients with clear consciousness and barrier-free communication; those who could offer complete pathological data; those who had no contraindication to MRI; those who had not received any treatment for TP before; those who volunteered to participate in the experiments.

Exclusion criteria included patients with psychiatric diseases; patients with complicated severe heart, liver, or kidney disorders; those who participated in other clinical experiments concurrently; pregnant or lactating women; those complicated with chronic obstructive pulmonary diseases.

### 2.2. Nursing Methods

The patients in the control group received routine nursing, which included basic drug treatment, daily nursing, and real-time monitoring of patients' vital signs.

Comprehensive nursing under the Omaha system was conducted for patients in the experimental group for three months. For data collection, the basic information of patients, such as age, gender, education, occupation, and family information, were collected. For health knowledge explanation, the professionally trained nursing staff explained the disease knowledge. They also formulated nursing plans and rehabilitation goals, let patients and their families understand self-nursing methods, and provide health guidance for the problems that patients may encounter after discharge from the hospital. Comprehensive nursing under the Omaha system was carried out on the physiology, psychology, and rehabilitation training of patients during hospitalization. In health, it was ensured that patients got enough sleep. A scientific diet was formulated according to their own conditions, which followed the principles of high protein, high vitamins, and high calories. The patients were instructed to avoid smoking and alcohol, eat more green vegetables and easily digestible foods, and take medication following the doctor's orders. Bad biological and dietary habits should be changed to improve immunity. In the physiological domain, patients who might experience physical discomfort such as pain during nursing were intervened. In the social psychological domain, communication with patients and their family members was made with a friendly attitude. The emotions such as great joy and great sadness should be avoided in patients, and the patients should be informed about the therapeutic nature of functional rehabilitation. The rush for success was inaccessible. Patients should build confidence in overcoming the disease and maintain an optimistic attitude. In rehabilitation training, passive training and active training were performed on the affected limbs of patients with stable conditions for paraplegia and muscle atrophy of the lower limbs. Joint flexion training was carried out 3–4 times a day, 10 minutes each time. Patients were assisted in doing upper limb activities, such as pulling pullers and lifting dumbbells that could exercise muscle strength of the upper limbs. Combined with naprapathy, massage, etc., muscle memory could be improved, giving full play to the body's metabolic function. In file management, nursing staff formulated a discharge rehabilitation plan according to the individual needs of patients and instructed patients and their families to train according to the rehabilitation plan.

### 2.3. MRI Examination Methods

3.0T multisource magnetic resonance instrument was used, with spine surface coil. The scanning range included SCI and compressed spots. Scanning parameters were set as follows. The routine sequences included fast spin echo (FES) sequence, sagittal T1-weighted imaging (T1WI), and sagittal T2-weighted imaging (T2WI). For FES and T1WI, the time of echo (TE) was 652 ms, and the time of repetition (TR) was 25 ms. For T2WI, TE was 3450 ms, while TR was 75 ms. The fat-suppression sequence was the short time inversion recovery (STIR) sequence, with TE of 2550 ms and TR of 80 ms. For diffusion-weighted imaging (DWI) sequence, TE, TR, the field of view, slice thickness, and slice interval were 3000 ms, 65 ms, 265 × 265 mm, 3.5 mm, and 3.5 mm, respectively.

### 2.4. Observation Indicators

#### 2.4.1. Basic Information

The gender, age, body mass index (BMI), causes of injury (traffic accident, injury by a heavy object, falling from a height, etc.), and the average course of disease were collected.

#### 2.4.2. Quality of Life

The quality of life was assessed by the Nottingham Health Profile-Quality of Life (NHP-QOL). The patient's energy, pain, condition, physical, social, and sleep indicators were evaluated. The higher the score, the worse the patient's quality of life.

#### 2.4.3. Nursing Outcomes

Nursing outcomes were assessed using the short form 36 (SF-36) health survey [17], which was composed of physical, psychological, environmental, and social health domains. The higher scores indicated better nursing outcomes.

#### 2.4.4. Caregiver Burden Survey

The Zarit Caregiver Burden Interview (ZBI) [18] consisted of a total of 22 items, each of which adopted a 4-point scale, with a maximum of 88 points. The higher the score, the heavier the caregiving burden. When the ZBI score was <20 points, 20–39 points, 40–59 points, and ≥60 points, the caregiving burden was assessed as no, mild, moderate, and severe, respectively.

#### 2.4.5. Comparison of Adverse Reactions

During the nursing period, the joint stiffness, muscle atrophy, pressure ulcer, and infection that occurred in the two groups of patients were observed and recorded.

#### 2.4.6. Imaging Parameter

The acquired MRI images were sent to the workstation for processing. The apparent diffusion coefficient (ADC) was measured at the most severely compressed spot of the spinal cord in the patients.

### 2.5. Statistical Methods

Statistical analysis of the data was made using SPSS 26.0. All measurement data were expressed as mean ± standard deviation. After the normality test, the data conforming to the normal distribution were compared between the two groups at different time points by a two-factor repeated-measurement analysis of variance (ANOVA). The comparisons between groups at the same time point were made by independent sample *t*-test. The comparison of each indicator within the same group at different time points was performed by one-way repeated-measurement ANOVA, and the least significant difference (LSD) method was adopted for the further pairwise comparisons. The data that did not conform to the normal distribution were compared between groups at different time points using generalized estimating equations, and further pairwise comparisons were also performed via the LSD method. The test standard of *P* < 0.05 indicated that the difference was of statistical significance.

## 3. Results

### 3.1. Comparison of Basic Data

The basic data of patients are compared between the experimental group and the control group in Figure 1. The number of males and females, age, BMI, causes of injury (traffic accident, injury by a heavy object, or falling from a height), and the average course of disease were not observably different between the two groups (*P* > 0.05).

### 3.2. MRI Findings

Figure 2 displays the MRI images of a 25-year-old male patient before and after intervention. For his vital signs, flaccid paralysis of both upper limbs was observed, muscle strength of both upper limbs was grade 1, tendon reflexes disappeared, pathological reflexes were not elicited, and gatism occurred. MRI showed intramedullary high signal and compression of the spinal cord on admission. Six months after discharge, MRI showed that the compression of the spinal cord was relieved and the dural sac was well filled.

Figure 3 presents the MRI images of a 52-year-old male patient before and after the nursing intervention. It was manifested as numbness and weakness of both upper limbs, aggravation of walking weakness, gatism, and pathological reflex disorders. On admission, MRI showed that the white lines of dural sac compression disappeared, and the spinal cord was compressed, with the abnormal intramedullary signal. Six months after discharge, it could be observed from MRI images that the dural sac compression was relieved, and the double white lines were restored, and there was no portal shaft rupture and portal closure.

### 3.3. Comparison of Scores of Quality of Life and Caregiving Burden

The comparison results of quality-of-life scores and caregiving burden scores of the two groups of patients at each time point are shown in Table 1. After being processed by the two-factor repeated-measurement ANOVA, the quality-of-life scores and caregiving burden scores of patients showed statistically significant differences in different groups, time points, and the interaction effect between groups and time points (*P* < 0.05).

The independent samples *t*-test showed that there was no significant difference in the quality-of-life scores and caregiving burden scores between groups at the same time point before discharge (*P* > 0.05). The scores of caregiving burden were greatly lower of the experimental group than those of the control group 3 months and 6 months after discharge, with differences of statistical significance (*P* < 0.05).

Through the one-way repeated-measurement ANOVA, significant differences were indicated in the quality-of-life scores and caregiving burden scores in the same groups but at different time points (*P* < 0.05). The LSD method was further used for pairwise comparing the scores between groups at different time points. The quality-of-life scores of both groups were remarkably higher 3 months and 6 months after discharge than those before discharge; those 6 months later were also remarkably higher than those 3 months after discharge, showing statistically significant differences (*P* < 0.05). The scores of caregiving burden before discharge were significantly higher than those 3 months and 6 months after discharge. In the experimental group, the caregiving burden scores 3 months after discharge were considerably higher than those 6 months after discharge; the differences were all statistically significant (*P* < 0.05).

### 3.4. Comparison of Nursing Outcome Scores in Environmental Domain

The comparison results of the health scores of the two groups of patients at each time point are listed in Table 2. After generalized estimating equation analysis, there were statistically significant differences in the health scores at different time points and in different groups (*P* < 0.05). There was not a significant difference in the interaction effect between grouping and time points (*P* > 0.05).

At the same time point, the health scores before discharge were not greatly different from those 3 months after discharge (*P* > 0.05). Those in the experimental group were extraordinarily higher than those in the control group 6 months after discharge, with differences of statistical significance (*P* < 0.05).

The health scores at different time points in the same groups suggested that the differences were statistically significant (*P* < 0.05). The LSD method was applied for pairwise comparisons of the health scores between the two groups at different time points. Three months and six months after discharge, the scores in both groups were markedly higher than those before discharge, and those six months after discharge were significantly higher than those 3 months after discharge in the experimental group; the differences were considered as statistically significant (*P* < 0.05).

### 3.5. Comparison of Psychosocial Scores

Table 3 shows the comparison results of scores of psychosocial domain between the two groups at each time point. Under generalized estimating equation analysis, the scores of social interactions, role change, mental health, and care of patients were statistically different at different time points, in different groups, and in the interaction effects of time points and groups (*P* < 0.05).

At the same time point, no significant difference was shown in the scores of social interactions, role change, mental health, and care between the two groups of patients before discharge (*P* > 0.05). The scores of social interactions had not shown a significant difference between the two groups 3 months after discharge (*P* > 0.05). The scores of role change, mental health, and care 3 months after discharge and the scores of all the 4 items 6 months after discharge were observably higher in the experimental group than those in the control group, showing differences of statistical significance (*P* < 0.05).

The analysis results of social interactions, role change, mental health, and care scores in the same groups were statistically different at different time points (*P* < 0.05). As the LSD method was adopted, the scores of these 4 items were further compared. Those scores 3 months and 6 months after discharge were significantly higher than those before discharge, and those after 6 months were also observably higher than those after 3 months; the differences were all statistically significant (*P* < 0.05).

### 3.6. Comparison of Physiological Scores at Each Time Point

The scores of the physiological domain in the two groups at each time point are shown in Table 4. The scores of oral hygiene, skin, neuromusculoskeletal (NMS) system, defecation function, urination function, and contagion/infection were analyzed by generalized estimating equations. These scores showed differences of statistical significance between groups, at different time points, and in the interaction between groups and corresponding time points (*P* < 0.05).

At the same time points, the scores of oral hygiene, skin, NMS system, defecation function, urination function, and contagion/infection were not significantly different between groups before discharge (*P* > 0.05). The scores of oral hygiene, skin, NMS, defecation function, urination function, and contagion/infection in the experimental group were distinctively higher than those in the control group 3 months and 6 months after discharge, with the statistically significant differences (*P* < 0.05).

In the same groups, the scores of oral hygiene, skin, NMS, defecation function, urination function, and contagion/infection were statistically different at different time points (*P* < 0.05). The scores of these 6 items were further compared with the LSD method at different time points between the two groups. The scores after discharge were significantly higher than before discharge, and those after 6 months were significantly higher than those after 3 months; all the differences were of statistical significance (*P* < 0.05).

### 3.7. Comparison of Health-Related Behavior Scores

The scores of the health-related behaviors of the two groups of patients at each time point are shown in Table 5. The scores of nutrition, healthcare supervision, and rest/sleep patterns were analyzed through the generalized estimating equations, from which there were statistically significant differences in the interaction effects between time points and corresponding groups, between groups, and at each time point (*P* < 0.05).

The scores of nutrition, healthcare supervision, and rest/sleep patterns showed no significant difference before discharge between the two groups at the same time point (*P* > 0.05). The scores of the three items in the experimental group were considerably higher than those in the control group 3 and 6 months after discharge, suggesting statistically significant differences (*P* < 0.05).

The scores of nutrition, healthcare supervision, and rest/sleep patterns at different time points were statistically different in the same groups (*P* < 0.05). The scores were compared pairwise between the two groups at different time points via the LSD method. These scores were markedly higher after discharge than those before discharge in both groups; meanwhile, those 6 months after discharge were also observably higher than those after 3 months; the differences were all statistically significant (*P* < 0.05).

### 3.8. Comparison of ADC Values

As shown in Figure 4, no statistically significant difference was found in the ADC values between the two groups of patients at admission (*P* > 0.05). The ADC values of both groups 6 months after discharge were substantially lower than those at admission, with differences of statistical significance (*P* < 0.05). The ADC value of patients in the experimental group 6 months after discharge (1.063 ± 0.148) was significantly lower than that in the control group (1.325 ± 0.245), which showed a difference in statistical significance (*P* < 0.05).

### 3.9. Complications in Patients in the Two Groups

There were 0 cases complicated with joint stiffness; 0 cases with muscle atrophy; 1 case with pressure ulcers; 1 case with infection in the experimental group, and 2, 1, 3, and 2 cases suffered from joint stiffness, muscle atrophy, pressure ulcers, and infection, respectively, in the control group. The incidence of complications in the experimental group (6.67%) was greatly lower than that in the control group (23.33%), showing a difference of statistical significance (*P* < 0.05) (Figure 5).

## 4. Discussion

TP is a clinical disease due to SCI or blood circulation disorder caused by external injury, and it is severe with a long treatment period. If the nursing and treatment are not in place, it will have a very serious impact on the quality of life and long-term prognosis of patients, greatly increasing the burden on families and society. Therefore, seeking an efficient rehabilitation nursing program is a hot topic in clinical research [19–21]. In total, 60 TP patients were included and divided into the experimental group with 30 cases treated with Omaha system-based comprehensive nursing and the control group with the other 30 cases that received routine nursing. All the objects were examined by MRI scanning. First, the basic data of the two groups of patients were compared, from which the number of males and females, age, BMI, causes of injury, and the average course of disease were not significantly different between the two groups (*P* > 0.05). Thus, feasibility for subsequent studies was provided. The scores of quality of life 3 months and 6 months after discharge in the experimental group were significantly higher than those in the control group. The scores of caregiving burden were observably lower than those in the control group, suggesting differences of statistical significance (*P* < 0.05). Quality of life refers to the evaluation of the physical, psychological, and social functions of individuals, that is, the quality of health. The quality of life of patients is also an important indicator of the effectiveness of the health nursing services they receive [22]. This research showed that the quality-of-life scores of the experimental group were significantly higher than those in the control group both 3 and 6 months after discharge; the differences were statistically significant (*P* < 0.05). Such a result proved that comprehensive nursing under the Omaha system could improve the quality of life of patients effectively compared with routine nursing. In addition, the caregiving burden scores of the experimental group were highly lower than those in the control group 3 months and 6 months after discharge, having the differences statistically significant (*P* < 0.05). This was similar to the findings of Jiang et al. [23]. Patients with TP have poor self-care ability and need careful long-term care from their families, especially patients with poor conditions. This will reduce their family members' expectations for future life. The results demonstrated that comprehensive nursing under the Omaha system could help patients improve their self-care ability and reduce the caregiving burden of family members effectively.

The nursing outcome scores in the environmental domain of patients were analyzed, from which no significant difference was shown between groups before discharge and 3 months after discharge (*P* > 0.05). The nursing outcome scores in the experimental group were significantly higher than those in the control group 6 months after discharge, and the differences were considered of statistical significance (*P* < 0.05). With the comprehensive nursing under the Omaha system, a corresponding rehabilitation plan could be formulated according to the individual situation of the patients, helping the patients to take exercise training reasonably, thereby improving the health issues for long-term staying in bed. Moreover, the role change, mental health, and care scores in the experimental group were memorably higher than those in the control group 3 and 6 months after discharge, going with the statistically significant differences (*P* < 0.05). It was indicated that the Omaha system-based comprehensive nursing could improve the psychological wellbeing of patients by keeping their body and mind happy and participating in family and social life. The scores of oral hygiene, skin, NMS, defecation function, urination function, and contagion/infection in the experimental group were also markedly higher than those in the control group 3 months and 6 months after discharge; the differences were statistically significant (*P* < 0.05). Through scientific and reasonable functional training, various physiological functions of patients were improved so as to help patients return to normal life as soon as possible. The result proved that compared with routine nursing, comprehensive nursing under the Omaha system could better promote the patients to recover physiological functions and improve the quality of daily life [24]. The scores of nutrition, healthcare supervision, and rest/sleep pattern in the experimental group were significantly higher as well than those in the control group 3 and 6 months after discharge, indicating statistically significant differences (*P* < 0.05). Thus, with comprehensive nursing under the Omaha system, a reasonable nutrient intake could be arranged to improve the sleep quality of patients.

The complications of the patients were followed up and recorded. In the experimental group, 0, 0, 1, and 1 cases got joint stiffness, muscle atrophy, pressure ulcers, and infection, respectively. In the control group, joint stiffness, muscle atrophy, pressure ulcers, and infection occurred in 2 cases, 1 case, 3 cases, and 2 cases, respectively. The incidence of complications in the experimental group was 6.67%, significantly lower than 23.33% in the control group (*P* < 0.05), indicating that comprehensive nursing under the Omaha system could reduce the incidence of complications in patients to improve the long-term prognosis. Besides, MRI was performed for examination on admission and 3 months after discharge. MRI showed that the white lines for the compression of the dural sac disappeared, the spinal cord was compressed, and the intramedullary signal turned out to be abnormal. Six months after discharge, MRI showed that the compression of the dural sac was relieved and the double white lines recovered. This suggested that the traumatic SCI of patients was greatly improved after nursing and treatment, and MRI could clearly assess the recovery of patients [25]. In quantitative evaluation, the ADC value of patients in the experimental group 6 months after discharge was remarkably lower than that in the control group, and the difference was shown of statistical significance (*P* < 0.05). The ADC value could evaluate the integrity of the white matter tract in the spinal cord; the smaller the value, the better the severer of SCI. The results illustrated that comprehensive nursing under the Omaha system could improve SCI in patients with TP effectively and promote the clinical treatment effect.

## 5. Conclusion

In this research, comprehensive nursing under the Omaha system was given in the treatment of 60 patients with TP, and MRI multisequence imaging scans were performed on the patients before and after treatment. Finally, it was proved that the Omaha system-based comprehensive nursing could effectively improve the clinical treatment effect of patients with SCI, reduce the incidence of complications, and promote the quality of life and nursing outcomes of patients. However, the sample size of the patients selected in this research was relatively small, the samples were from a single source, and the postoperative follow-up time was short. A wider range of case data would be included in the future study, and the clinical treatment means of TP would be discussed more in depth. All in all, this research had a great guiding significance in the nursing and treatment of TP patients.

## Figures and Tables

**Figure 1:** Comparison of the basic data of patients in the two groups. The comparisons of (a) gender, (b) age and BMI, (c) causes of injury, and (d) the average course of the disease. (1) Traffic accidents, (2) injury by a heavy object, and (3) falling from a height.

**Figure 2:** MRI manifestations of a male patient before and after the intervention. The patient was 25 years old and admitted to hospital 3 days after neck and shoulder pain and limb weakness caused by a heavy object hitting the neck. (a) Before the intervention. (b) After the intervention.

**Figure 3:** MRI images of a male patient before and after the intervention. The patient was 52 years old, with lumbar pain, numbness, and weakness of both upper limbs due to contusions and was admitted to the hospital for aggravation of walking weakness for 3 months. (a) Before the intervention. (b) After intervention.

**Figure 4:** Comparison of ADC values between groups before and after the nursing intervention.  ^*∗*^Compared with the values on admission, *P* < 0.05; # compared with the experimental group, *P* < 0.05.

**Figure 5:** Complications of patients in the two groups. (a) The number of cases with joint stiffness, muscle atrophy, pressure ulcers, and infections; (b) the incidence of complications in two groups. 1–4 represented joint stiffness, muscle atrophy, pressure ulcers, and infections, respectively. #Compared with the incidence of the experimental group, *P* < 0.05.

**Table 1:** Quality-of-life scores and caregiving burden scores between groups at each time point $\left(\bar{x}\pm s\right)$.

Indicators	Time points	Experimental group (*n* = 30)	Control group (*n* = 30)	*t*	*P*
Quality-of-life scores	Before discharge	283.40 ± 3.38	282.70 ± 2.45	0.918	0.362
	3 months after discharge	302.30 ± 3.29^a^	292.80 ± 3.45^a^	10.915	<0.001
	6 months after discharge	305.20 ± 2.77^ab^	297.97 ± 3.44^ab^	8.970	<0.001
	*F*	391.999	297.284	—	—
	*P*	<0.001	<0.001	—	—

Caregiving burden scores	Before discharge	60.77 ± 5.22	60.33 ± 5.22	0.321	0.749
	3 months after discharge	48.67 ± 6.97^a^	52.83 ± 6.37^a^	2.416	0.019
	6 months after discharge	43.40 ± 4.97^ab^	50.07 ± 7.14^a^	4.197	<0.001
	*F*	64.556	20.231	—	—
	*P*	<0.001	<0.001	—	—

Notes: time point F (quality-of-life score) = 678.172, *P* < 0.001; F grouping (quality-of-life score) = 116.678, *P* < 0.001; the interaction between F grouping and time point F (quality-of-life score) = 37.258, *P* < 0.001. Time point F (caregiving burden score) = 77.029, *P* < 0.001; F grouping (caregiving burden score) = 17.427, *P* < 0.001; the interaction between F grouping and time point F (caregiving burden score) = 4.945, *P* = 0.009. ^a^Compared with those before discharge. ^b^Compared with those 3 months after discharge, *P* < 0.05.

**Table 2:** Comparison of health scores of patients between groups at each time point $\left(\bar{x}\pm s\right)$.

Time points	Experimental group (*n* = 30)	Control group (*n* = 30)	*Waldχ* ^2^	*P*
Before discharge	6.23 ± 0.90	6.13 ± 0.90	0.192	0.661
3 months after discharge	10.47 ± 1.11^a^	10.33 ± 1.03^a^	0.242	0.623
6 months after discharge	11.43 ± 1.01^ab^	10.70 ± 1.06^a^	7.849	0.005
*Waldχ * ^2^	590.622	408.478	—	—
*P*	<0.001	<0.001	—	—

Notes: Wald*χ*^2^ time point = 971.012, *P* < 0.001; Wald*χ*^2^ grouping = 4.580, *P* = 0.032; the interaction between Wald*χ*^2^ grouping and Wald*χ*^2^ time point = 3.766, *P* = 0.152. a and b represented that *P* < 0.05 compared with those before discharge and 3 months after discharge, respectively.

**Table 3:** Comparison of psychosocial scores between groups at each time point $\left(\bar{x}\pm s\right)$.

Indicators	Time points	Experimental group (*n* = 30)	Control group (*n* = 30)	*Waldχ* ^2^	*P*
Social interactions	Before discharge	5.27 ± 1.08	5.33 ± 0.88	0.071	0.790
	3 months after discharge	8.43 ± 1.10^a^	8.10 ± 0.92^a^	1.665	0.197
	6 months after discharge	11.83 ± 0.99^ab^	10.27 ± 1.11^ab^	34.498	<0.001
	*Waldχ* ^2^	658.662	502.014	—	—
	*P*	<0.001	<0.001	—	—

Role change	Before discharge	5.60 ± 0.56	5.53 ± 0.82	0.140	0.709
	3 months after discharge	9.53 ± 0.97^a^	7.20 ± 0.89^a^	97.480	<0.001
	6 months after discharge	10.93 ± 1.08^ab^	8.53 ± 1.04^ab^	79.347	<0.001
	*Waldχ* ^2^	878.787	148.942	—	—
	*P*	<0.001	<0.001	—	—

Mental health	Before discharge	7.13 ± 0.94	7.17 ± 0.83	0.022	0.882
	3 months after discharge	10.7 ± 1.29^a^	8.07 ± 1.05^a^	77.850	<0.001
	6 months after discharge	12.17 ± 0.99^ab^	10.23 ± 0.86^ab^	67.914	<0.001
	*Waldχ* ^2^	358.556	236.849	—	—
	*P*	<0.001	<0.001	—	—

Care	Before discharge	8.23 ± 0.86	8.27 ± 1.08	0.018	0.893
	3 months after discharge	11.27 ± 1.05^a^	10.20 ± 0.96^a^	17.455	<0.001
	6 months after discharge	13.27 ± 0.91^ab^	11.23 ± 1.04^ab^	67.369	<0.001
	*Waldχ* ^2^	491.071	137.016	—	—
	*P*	<0.001	<0.001	—	—

Notes: Wald*χ*^2^ time point (social interactions) = 1096.086, *P* < 0.001; Wald*χ*^2^ grouping (social interactions) = 14.151, *P* < 0.001; the interaction between Wald*χ*^2^ grouping and Wald*χ*^2^ time point (social interactions) = 20.568, *P* < 0.001. Wald*χ*^2^ time point (role change) = 768.170, *P* < 0.001; Wald*χ*^2^ grouping (role change) = 134.883, *P* < 0.001; the interaction between Wald*χ*^2^ grouping and Wald*χ*^2^ time point (role change) = 81.906, *P* < 0.001. Wald*χ*^2^ time point (mental health) = 559.248, *P* < 0.001; Wald*χ*^2^ grouping (mental health) = 113.148, *P* < 0.001; the interaction between Wald*χ*^2^ grouping and time point (mental health) = 61.177, *P* < 0.001. Wald*χ*^2^ time point (care) = 551.096, *P* < 0.001; Wald*χ*^2^ grouping (care) = 46.083, *P* < 0.001; the interaction between Wald*χ*^2^ grouping and time point (care) = 36.296, *P* < 0.001. ^a^Compared with the scores before discharge, *P* < 0.05. ^b^Compared with the scores 3 months after discharge, *P* < 0.05.

**Table 4:** Comparison of physiological scores between two groups at each time point $\left(\bar{x}\pm s\right)$.

Indicators	Time points	Experimental group (*n* = 30)	Control group (*n* = 30)	*Waldχ* ^2^	*P*
Oral hygiene	Before discharge	7.73 ± 1.17	7.57 ± 1.07	0.341	0.559
	3 months after discharge	10.37 ± 1.10^a^	8.70 ± 0.75^a^	48.765	<0.001
	6 months after discharge	12.9 ± 1.03^ab^	9.23 ± 0.94^ab^	215.815	<0.001
	*Waldχ* ^2^	476.260	64.713	—	—
	*P*	<0.001	<0.001	—	—

Skin	Before discharge	7.23 ± 0.77	7.17 ± 0.99	0.088	0.767
	3 months after discharge	11.23 ± 1.17^a^	9.37 ± 0.96^a^	47.276	<0.001
	6 months after discharge	14.07 ± 0.64^ab^	11.23 ± 1.72^ab^	74.306	<0.001
	*Waldχ* ^2^	1897.736	128.608	—	—
	*P*	<0.001	<0.001	—	—

NMS	Before discharge	7.33 ± 0.88	7.37 ± 0.96	0.020	0.887
	3 months after discharge	10.37 ± 0.89^a^	9.30 ± 0.75^a^	26.078	<0.001
	6 months after discharge	12.63 ± 0.85^ab^	10.77 ± 1.17^ab^	51.978	<0.001
	*Waldχ* ^2^	649.053	162.647	—	—
	*P*	<0.001	<0.001	—	—

Defecation function	Before discharge	7.93 ± 1.08	8.03 ± 1.16	0.124	0.725
	3 months after discharge	11.23 ± 0.90^a^	9.57 ± 0.68^a^	68.058	<0.001
	6 months after discharge	13.83 ± 0.91^ab^	11.37 ± 0.93^ab^	111.452	<0.001
	*Waldχ* ^2^	656.504	253.275	—	—
	*P*	<0.001	<0.001	—	—

Urination function	Before discharge	7.63 ± 0.96	7.73 ± 1.02	0.158	0.691
	3 months after discharge	10.17 ± 0.83^a^	9.57 ± 1.10^a^	5.834	0.016
	6 months after discharge	13.53 ± 1.01^ab^	11.27 ± 1.36^ab^	55.488	<0.001
	*Waldχ* ^2^	509.658	131.380	—	—
	*P*	<0.001	<0.001	—	—

Contagion/infection	Before discharge	7.23 ± 0.97	7.13 ± 0.86	0.184	0.668
	3 months after discharge	11.33 ± 1.27^a^	9.93 ± 0.87^a^	25.739	<0.001
	6 months after discharge	12.97 ± 0.85^ab^	10.63 ± 1.25^ab^	74.317	<0.001
	*Waldχ* ^2^	594.236	203.727	—	—
	*P*	<0.001	<0.001	—	—

Notes: Wald*χ*^2^ time point (oral hygiene) = 471.340, *P* < 0.001; Wald*χ*^2^ grouping (oral hygiene) = 119.670, *P* < 0.001; the interaction between Wald*χ*^2^ grouping and time point (oral hygiene) = 129.778, *P* < 0.001. Wald*χ*^2^ time point (skin) = 709.896, *P* < 0.001; Wald*χ*^2^ grouping (skin) = 103.890, *P* < 0.001; the interaction between Wald*χ*^2^ grouping and corresponding time point (skin) = 49.930, *P* < 0.001. Wald*χ*^2^ time point (NMS) = 662.095, *P* < 0.001; Wald*χ*^2^ grouping (NMS) = 51.130, *P* < 0.001; the interaction between Wald*χ*^2^ grouping and Wald*χ*^2^ time point (NMS) = 31.678, *P* < 0.001. Wald*χ*^2^ time point (defecation function) = 873.504, *P* < 0.001; Wald*χ*^2^ grouping (defecation function) = 74.332, *P* < 0.001; the interaction between Wald*χ*^2^ grouping and time point (defecation function) = 64.897, *P* < 0.001. Wald*χ*^2^ time point (urination function) = 508.117, *P* < 0.001; Wald*χ*^2^ grouping (urination function) = 40.045, *P* < 0.001; the interaction between Wald*χ*^2^ grouping and Wald*χ*^2^ time point (urination function) = 32.742, *P* < 0.001. Wald*χ*^2^ time point (contagion/infection) = 704.296, *P* < 0.001; Wald*χ*^2^ grouping (contagion/infection) = 60.177, *P* < 0.001; the interaction between Wald*χ*^2^ grouping and Wald*χ*^2^ time point (contagion/infection) = 37.187, *P* < 0.001. ^a^Compared with the scores before discharge, *P* < 0.05. ^b^Compared with the scores 3 months after discharge, *P* < 0.05.

**Table 5:** Comparison of health-related behavior scores between groups at different time points $\left(\bar{x}\pm s\right)$.

Indicators	Time points	Experimental group (*n* = 30)	Control group (*n* = 30)	*Waldχ* ^2^	*P*
Nutrition	Before discharge	7.03 ± 1.03	7.10 ± 0.89	0.075	0.790
	3 months after discharge	11.37 ± 1.00^a^	9.03 ± 0.96^a^	87.604	<0.001
	3 months after discharge	13.63 ± 0.89^ab^	11.03 ± 1.22^ab^	92.275	<0.001
	*Waldχ* ^2^	786.625	166.960	—	—
	*P*	<0.001	<0.001	—	—

Healthcare supervision	Before discharge	6.23 ± 0.94	6.07 ± 0.91	0.508	0.476
	3 months after discharge	9.67 ± 1.16^a^	9.00 ± 0.79^a^	7.059	0.008
	3 months after discharge	12.87 ± 0.86^ab^	11.17 ± 1.34^ab^	35.324	<0.001
	*Waldχ* ^2^	747.824	385.661	—	—
	*P*	<0.001	<0.001	—	—

Rest/sleep pattern	Before discharge	7.13 ± 0.82	7.03 ± 0.85	0.223	0.637
	3 months after discharge	10.33 ± 1.16^a^	8.17 ± 0.79^a^	74.340	<0.001
	3 months after discharge	13.07 ± 0.98^ab^	9.87 ± 0.73^ab^	212.677	<0.001
	*Waldχ* ^2^	630.754	181.204	—	—
	*P*	<0.001	<0.001	—	—

Notes: Wald*χ*^2^ time point (nutrition) = 763.957, *P* < 0.001; Wald*χ*^2^ grouping (nutrition) = 141.041, *P* < 0.001; the interaction between Wald*χ*^2^ grouping and time point (nutrition) = 64.067, *P* < 0.001. Wald*χ*^2^ time point (healthcare supervision) = 1046.382, *P* < 0.001; Wald*χ*^2^ grouping (healthcare supervision) = 24.399, *P* < 0.001; the interaction between Wald*χ*^2^ group and time point (healthcare supervision) = 17.758, *P* < 0.001. Wald*χ*^2^ time point (rest/sleep pattern) = 758.333, *P* < 0.001; Wald*χ*^2^ grouping (rest/sleep pattern) = 180.107, *P* < 0.001; the interaction between Wald*χ*^2^ grouping and Wald*χ*^2^ time point (rest/sleep pattern) = 102.302, *P* < 0.001. ^a^Compared with the scores before discharge, *P* < 0.05. ^b^Compared with the scores 3 months after discharge, *P* < 0.05.

## Data Availability

The data used to support the findings of this study are available from the corresponding author upon request.

## References

[1] Gupta N. (2020 Mar 11). Recommendations for standards of physiotherapy care following complete traumatic paraplegia in India. *Spinal Cord Ser Cases*.

[2] Brunelli G. (2005). Research on the possibility of overcoming traumatic paraplegia and its first clinical results. *Current Pharmaceutical Design*.

[3] Wang H. (1992 Dec). A survey of the treatment of traumatic paraplegia by traditional Chinese medicine. *Journal of Traditional Chinese Medicine*.

[4] Byra S. (2019 Apr). Basic hope and posttraumatic growth in people with traumatic paraplegia- the mediating effect of acceptance of disability. *Spinal Cord*.

[5] Donovan W. H., Dwyer A. P. An update on the early management of traumatic paraplegia (nonoperative and operative management). *Clinical Orthopaedics and Related Research*.

[6] Rahimi M., Torkaman G., Ghabaee M., Ghasem-Zadeh A. (2020 Jan). Advanced weight-bearing mat exercises combined with functional electrical stimulation to improve the ability of wheelchair-dependent people with spinal cord injury to transfer and attain independence in activities of daily living: a randomized controlled trial. *Spinal Cord*.

[7] Bohler J. Die behandlung traumatisch querschnittsgelähmter [treatment of traumatic paraplegia]. *Wiener Klinische Wochenschrift*.

[8] Dick T. B. (1969 Nov). Traumatic paraplegia pre-Guttmann. *Paraplegia*.

[9] Owolabi L. F., Ibrahim A., Samaila A. A. (2011 Apr-Jun). Profile and outcome of non-traumatic paraplegia in Kano, northwestern Nigeria. *Annals of African Medicine*.

[10] Xie S. X., Yu Z. C., Lv Z. H. (2021 Jan). Multi-disease prediction based on deep learning: a survey. *Computer Modeling in Engineering and Sciences*.

[11] Evangelista Santos Barcelos A. C., Scardino F. B., Patriota G. C., Rotta J. M., Botelho R. V. (2009 Apr). Paraparesis or incomplete paraplegia? How should we call it?. *Acta Neurochirurgica*.

[12] Yu Z. C., Amin S. U., Alhussein M., Lv Z. H. (2021 Feb). Research on disease prediction based on improved DeepFM and IoMT. *IEEE Access*.

[13] Hu M., Zhong Y., Xie S., Lv H., Lv Z. (2021 Jul 30). Fuzzy system based medical image processing for brain disease prediction. *Frontiers in Neuroscience*.

[14] Gbadamosi H., Mensah Y. B., Asiamah S. (2018 Sep). MRI features in the non-traumatic spinal cord injury patients presenting at the Korle Bu Teaching Hospital. *Accra. Ghana Med J*.

[15] Musubire A. K., Meya D. B., Katabira E. T. (2019 Jan 15). Epidemiology of non-traumatic spinal cord injury in Uganda: a single center, prospective study with MRI evaluation. *BMC Neurology*.

[16] Wiklund I. (1990). The Nottingham Health Profile--a measure of health-related quality of life. *Scandinavian Journal of Primary Health Care - Supplement*.

[17] Brazier J. E., Harper R., Jones N. M. (1992). Validating the SF-36 health survey questionnaire: new outcome measure for primary care. *BMJ*.

[18] Yu Y., Liu Z. W., Li T. X. (2020 Apr 6). A comparison of psychometric properties of two common measures of caregiving burden: the family burden interview schedule (FBIS-24) and the Zarit caregiver burden interview (ZBI-22). *Health and Quality of Life Outcomes*.

[19] Fattal C., Fabbro M., Rouays-Mabit H., Verollet C., Bauchet L. (2011 Jan). Metastatic paraplegia and functional outcomes: perspectives and limitations for rehabilitation care. Part 2. *Archives of Physical Medicine and Rehabilitation*.

[20] Niedeggen A., Giesecke J., Diederichs W., Bötel U. (1997 Aug). Die traumatische Querschnittlähmung. Möglichkeiten von Therapie und Rehabilitation an einem modernen Behandlungszentrum [Traumatic paraplegia. Possibilities of therapy and rehabilitation in a modern treatment center]. *Z Arztl Fortbild Qualitatssich*.

[21] Robinson D. M., Bazzi M. S., Millis S. R., Bitar A. A. (2018 Jul). Predictors of readmission to acute care during inpatient rehabilitation for non-traumatic spinal cord injury. *J Spinal Cord Med*.

[22] Denis A. R., Feldman D., Thompson C., Mac-Thiong J. M. (2018 May). Prediction of functional recovery six months following traumatic spinal cord injury during acute care hospitalization. *J Spinal Cord Med*.

[23] Jiang L., Sun L., Meng Q. (2021 Oct 29). Identification and relationship of quality of life and self-care ability among Chinese patients with traumatic spinal cord injuries: a cross-sectional analysis. *Brazilian Journal of Medical and Biological Research*.

[24] Wuermser L. A., Ho C. H., Chiodo A. E., Priebe M. M., Kirshblum S. C., Scelza W. M. (2007 Mar). Spinal cord injury medicine. 2. Acute care management of traumatic and nontraumatic injury Erratum in. *Archives of Physical Medicine and Rehabilitation*.

[25] Ueyama T., Tamaki N., Kondoh T., Miyamoto H., Akiyama H., Nagashima T. (1999 Aug). Non-traumatic acute paraplegia associated with cervical disc herniation: a case report. *Surgical Neurology*.

